# The Significance of Three-Dimensional Team Management in the Medical Community Model for Patients with Hypertension and Diabetes

**DOI:** 10.1155/2022/1960030

**Published:** 2022-04-11

**Authors:** Xiaoli Lu, Hualiang Tang, Tan Xu, Xuehui Song, Fei Jiang, Xie Zheng, Yang Li

**Affiliations:** ^1^Department of Cardiology, Anji People's Hospital, Anji 313300, China; ^2^Department of Cardiology, the First Affiliated Hospital of Baotou Medical College, I, nner Mongolia University of Science and Technology, Baotou 014010, China; ^3^Child Health Section, Anji Changshuo Street Health Center, Anji 313300, China; ^4^Department of Endocrinology,People's Hospital, Anji 313300, China

## Abstract

Diabetes and hypertension are the most common diseases and often coexist. Currently, hypertension is the most widespread chronic disease in China. To explore the value of three-dimensional team management in improving the effect of the management of primary diabetes and hypertension in patients in the medical community model, the expert team at the Department of Cardiology and Endocrinology of Anji County People's Hospital is selected to train 59 community general practitioners in the medical community model (the study group adopts the three-dimensional team management model in the medical community model), and another 59 community medical general practitioners adopts the conventional training method (the control group). The two groups of doctors managed patients with diabetes and hypertension who are registered in the jurisdiction (200 patients per group) as per the respective training methods. The three-dimensional management of the team under the medical community model significantly improves the diagnostic and treatment capabilities of grassroot general practitioners to better control patients' diabetes and hypertension levels.

## 1. Introduction

Population aging and rapid economic development have led to changes in behavior and lifestyle, and the prevalence of chronic diseases, such as diabetes, has increased rapidly. Diabetes has become a persistent public problem affecting the health of the Chinese population. Diabetes is a chronic, non-communicable disease that requires lifelong control and is often associated with hypertension [1]. Insulin resistance plays a vital role in the pathogenesis of diabetes and hypertension. Most diabetic patients have insulin resistance, and approximately 50% of hypertensive patients are also insulin resistant [2]. Therefore, the management of diabetes has changed from single blood glucose management to the comprehensive control of blood glucose and blood pressure. Actively performing standardized management of diabetic patients is a key measure to improve the level of blood glucose control [3].

In China, community health service centers are basic units to manage chronic diseases, such as diabetes and hypertension, and it is essential to evaluate the effects of relevant interventions [4]. Community medical personnel are indispensable in the prevention and treatment of diabetes and hypertension at the grassroot level. The concepts of diabetes and hypertension prevention, clinical knowledge, and practical abilities of community doctors are closely related to the disease control rate [5]. We established a chronic disease management team under the medical community model, targeted training grassroot community doctors, compared doctors' mastery of hypertension and diabetes-related knowledge before and after training, and discussed the value of three-dimensional team management under the medical community model to improve the management of grassroot diabetes and hypertension patients.

## 2. Materials and Methods

### 2.1. Study Information and Participant Selection

The research was conducted from January 2018 to July 2020, and the expert team at the Department of Cardiovascular Medicine and Endocrinology in Anji County People's Hospital is selected to train 59 community general practitioners in the medical community (the research group adopts the three-dimensional management of the team under the medical community model), and the other 59 community general practitioners adopt the conventional training method (the control group). The inclusion criteria as follows: (1) the age range of community doctors is 28–55 years old; (2) the titles of doctors participating in the training are primary and intermediate; (3) training is conducted in strict accordance with the training requirements, and 200 patients with type 2 diabetes or hypertension are managed by community doctors in each group; (4) the research program is approved by the Medical Ethics Committee. Exclusion criteria: (1) personnel who cannot participate in training on time and according to regulations; (2) doctors who have not yet obtained the required title; (3) specialists; (4) managed patients with hypertension and diabetes combined with major diseases of other systems.

The research proposal and related materials shall be provided after the medical ethics committee has studied and determined the disease and issued a document (hospital ethics approval 18).

### 2.2. Training Methods for Community Doctors

#### 2.2.1. Control Group (Conventional Training Methods in Adopting the Centralized Teaching Training Model)

Each community doctor received at least 6 h of diabetes and hypertension diagnoses and treatment knowledge training, annually. The training is mainly conducted by experts from municipal and district chronic disease prevention and control centers through large lectures.

#### 2.2.2. Study Group (Application of Three-Dimensional Team Management in the Medical Community Model)

This group included city and district chronic disease prevention and control hospital experts who inspected the community health service center quarterly, identified the problem, selected a typical case, and offered discussion-based on-site teaching and training. Furthermore, face-to-face counseling occurred with community doctors to teach, highlight the importance of health education, provide lifestyle treatment, promote knowledge about hypertension and diabetes, guide rational drug combination, and optimize treatment plans for patients with complications. The goal is to improve the diagnostic and treatment skill levels of responsible doctors in regional primary communities, establish an efficient chronic disease management team, strengthen the education of patients, including drug and nondrug treatment, and provide emotional management; this helped to better manage blood pressure and blood glucose, develop a healthy lifestyle, and improve quality of life. Each community doctor received on-site teaching training no less than six times for no less than 1 h each time.

### 2.3. Survey Indicators

Evaluations of community general practitioners' skills to diagnose and treat hypertension diseases follow the “Guidelines for the Prevention and Treatment of Hypertension in China [6],” and mainly investigate whether general practitioners can respond with accurate answers regarding the diagnosis and treatment of hypertension (blood pressure level classification, risk stratification, and antihypertensive treatment strategy), nondrug treatment strategy for hypertension (reasonable diet, weight control, physical exercise, smoking cessation, and balance psychology), and knowledge of hypertension drug treatment (syndrome of prudent use of diuretics, syndrome of prudent use/prohibition of *ß* blockers, syndrome of prohibition of angiotensin-converting enzyme inhibitor (ACEI) drugs, and syndrome of prudent use/prohibition of compound preparations).

The evaluation of community doctors' abilities to diagnose and treat diabetes is mainly based on the “practical goals and treatment of type 2 diabetes” [7] and the standards in the 2004 edition of “Guidelines for the Prevention and Treatment of Diabetes in China [8].” This involves the diagnosis of diabetes (diagnosis of type 2 diabetes, impaired glucose tolerance, and impaired fasting blood glucose), basic knowledge of diabetes (glycosylated hemoglobin (HbA1c) purpose, dyslipidemia characteristics, and blood glucose control objectives), and drug therapy knowledge (preferred drugs for obese patients and preferred drugs for nonobese patients) [9].

### 2.4. Observation Indicators for Patients with Hypertension and Diabetes

The fasting plasma glucose (FPG), postprandial 2 h blood glucose (2 hPG), glycosylated hemoglobin (HbA1c), 24 h average systolic blood pressure (SBP), 24 h average diastolic blood pressure (DBP), and medication compliance of patients with diabetes and hypertension managed by general practitioners in the two groups are compared after training [10].

All patients fasted for 12 h, and morning fasting elbow venous blood (5 ml) is taken. A Hitachi 7180 automatic biochemical analyzer glucose oxidase method is used to determine FPG and 2hPG, using high-pressure liquid chromatography to determine glycosylated hemoglobin HbA1c.

All patients received 24 h ambulatory blood pressure monitoring ([manufacturer: Aicanfi; model: ACF-D1] SBP, DBP, cuff 12 cm × 22 cm), with the instrument fixed onto the patient's right or left upper arm; daytime is set to 7 : 00–21 : 00, blood pressure measurement time interval is 20 min/time, night time is set to 21 : 00–7:00, time interval is 40 min/time, and monitoring times are > 80% for effective monitoring [11].

A questionnaire survey with newly admitted patients included questions on their basic situation, related information, and compliance evaluation [12]. Compliance evaluation is mainly conducted from four aspects: medication, diet, exercise, blood glucose, or blood pressure monitoring [13]. There are 15 questions in total. The score range for each question is 1–5 points. The higher the score, the higher the patient's compliance management. Scores ranging from 61 to 75 indicated good compliance, 46–60 are general compliance, and ≤45 are poor compliance.

### 2.5. Statistical Processing

We tested patients' FPG, 2hPG, and HbA1c values by normal distribution, which accorded with the approximate normal distribution or normal distribution, and are expressed as $\left(\bar{x}\pm s\right)$. The LSD-t test is used to compare the two groups. Counting data are expressed as percentages, non-grade comparison is performed using the *χ*2 test, and grade comparison between groups is performed using the Mann-Whitney *U* test. SPSS (version 21.0) is used for data processing, and the inspection level *a* is set at 0.05.

## 3. Experimental Results

### 3.1. Comparison of the Basic Situation of General Practitioners in the Study Group and the Control Group

The age, gender, professional title, and educational level are compared between the study group and the control group, and the difference is not statistically significant (*p* > 0.05).  Table 1 is the comparison of the basic situation of general practitioners in the study group and the control group.

### 3.2. Comparison of the Ability of General Practitioners in the Study Group and the Control Group to Diagnose and Treat Diabetes before and after Training

Before training, the correct response rates of type 2 diabetes diagnosis, impaired glucose tolerance, impaired fasting blood glucose, HbA1c purpose, dyslipidemia characteristics, blood glucose control objectives, preferred drugs for obese patients, and preferred drugs for nonobese patients are compared between the study group and the control group, and the difference is not statistically significant (*p* > 0.05). After training, the correct response rate of doctors in the study group to the diagnosis of type 2 diabetes, impaired fasting blood glucose, HbA1c purpose, dyslipidemia characteristics, blood glucose control objectives, and preferred drugs for obese patients is significantly higher than that in the control group, and the difference is statistically significant (*p* < 0.05).  Table 2 is the comparison of diabetes diagnosis and treatment ability before and after training.

### 3.3. Comparison of the Ability of General Practitioners in the Study Group and the Control Group to Diagnose and Treat Hypertension before and after Training

Before training, the correct response rates of blood pressure level classification, risk stratification, antihypertensive treatment strategy, reasonable diet, weight control, physical exercise, smoking cessation, balance psychology, careful use of diuretics, careful use/prohibition of beta blockers, ACEI drug prohibition, and careful use/prohibition of compound preparations are compared between the study group and the control group, and the difference is not statistically significant (*p* > 0.05). After training, the correct response rates of doctors in the study group on blood pressure level classification, antihypertensive treatment strategy, balance psychology, *ß*-blocker cautious/forbidden certificate, and compound preparation cautious/forbidden certificate are significantly higher than those in the control group, and the difference is statistically significant (*p* < 0.05).  Table 3 is the comparison of the ability to diagnose and treat hypertension before and after training.

### 3.4. Comparison of Baseline Data of Patients in the Study Group and the Control Group Intervened by General Practitioners

General practitioners in the study group and the control group intervened 200 patients with diabetes and hypertension, respectively. The baseline data of the two groups are compared, and the differences are not statistically significant (*p* > 0.05).  Table 4 is the comparison of baseline data of patients in the study group and the control group with general practitioner intervention.

### 3.5. The Blood Pressure Control of Patients in the Study Group and the Control Group

There are 100 patients with hypertension in the study group and 109 patients with hypertension in the control group. The SBP and DBP before intervention are compared between the study group and the control group, and the differences are not statistically significant (*P* > 0.05). After intervention, SBP in the study group is lower than that in the control group, and the difference is significant (*p* < 0.05).  Table 5 shows the blood pressure control status of study group and control group.

### 3.6. The Blood Glucose Control of the Study Group and the Control Group

There are 100 patients with diabetes in the study group and 91 patients with diabetes in the control group. The FPG, 2hPG, and HbA1c are compared between the study group and the control group before intervention, and the differences are not statistically significant (*p* > 0.05). After intervention, 2hPG and HbA1c in the study group are lower than those in the control group, and the difference is significant (*p* < 0.05).  Table 6 shows the blood sugar control status of the study group and the control group.

### 3.7. Comparison of Compliance between the Study Group and the Control Group

The complete compliance rate of the study group is 67.00%, the general rate is 27.00%, and the poor compliance rate is 6.00%. The complete compliance rate of the control group is 52.50%, the general rate is 35.50%, and the poor compliance rate is 12.00%. The difference between the two groups is significant (*p* < 0.05).  Table 7 is the comparison of compliance between the study group and the control group.

## 4. Analysis and Discussion

Because diabetes and hypertension are chronic diseases with a hidden onset, long course of disease, and need lifelong treatment, their prevention and treatment must be undertaken by most primary medical institutions, especially community health service centers, as well as primary and community doctors. Comprehensive community intervention has become important to treat chronic diseases at the grassroot level in China. The main problems are that management is not standardized, personalized disease management plans are lacking, and measures for different groups and individuals differ. To ensure that most primary chronic diseases are reasonably diagnosed and treated in community health service centers, it is necessary to improve the diagnosis and treatment skill levels of community doctors. Community doctors urgently need to update ideas as well as supplement knowledge and improve their skills to meet the growing needs for cardiovascular disease prevention and control in China.

We established a chronic disease management team under the medical community model to conduct targeted training for community doctors. To effectively reduce the incidence of mortality through cardiovascular diseases in the region, mastery of hypertension and diabetes-related knowledge and the changes in patients' related indicators before and after doctors' training are compared. The results revealed that after training, the study group doctors' correct response rates are significantly higher than the control group's (*p* < 0.05) to diagnose type 2 diabetes, impaired fasting blood glucose, dyslipidemia characteristics, blood glucose control objectives, and the preferred drugs for obese patients. The study group doctors' response rates for correctly classifying blood pressure levels, antihypertensive treatment strategies, balance psychology, *ß*-receptor blocker' caution/prohibition card, and compound preparations' caution/prohibition cards are significantly higher than the control group's (*p* < 0.05). After conducting three-dimensional team management training in the medical community model, the doctors' hypertension knowledge, case diagnosis, and abilities to treat are significantly higher than that of community doctors with conventional training.

According to the analysis, the main characteristics of the three-dimensional team management in the medical community model are cultivating the ability to diagnose accurately and providing effective treatment as the main goals. Other achievements include implementing face-to-face discussion, using interaction training methods, incorporating theory with practice, and ensuring pertinence and practicability. The teacher is an expert, rich in clinical and teaching experience, from city and district chronic disease prevention and control hospitals; thus, common cases are used to introduce the problems that community doctors often encounter in diagnosing and treating such cases. Teachers guide students by discussing these problems; thereafter, they gradually explain the knowledge relevant to the case and finally return to the case and the problem so that the students can truly master the diagnosis and treatment methods of such cases. The entire training process encouraged students' learning initiatives, made an impression, and is easy to accept.

After the intervention, the study group's SBP, 2hPG, and HbA1c levels are significantly lower than the control group's (*p* < 0.05). Hence, three-dimensional team management under the medical community model can strengthen patients' self-management abilities and indirectly affect patients' laboratory test indexes. Through health education, patients are guided to strictly follow the doctor's advice and take correct dosages of medicines timeously so that FPG, 2hPG, HbA1c, and other indicators are gradually decreased and normalized. The compliance rate of the study group is significantly better than the control group (*p* < 0.05). This shows that the three-dimensional management of the team under the medical community model has a high application value and can effectively improve the quality of family management as well as the effect of disseminating disease knowledge and service satisfaction. Family intervention and treatment methods can help educate patients to develop healthy living habits while formulating detailed and reasonable treatment plans, fully using various family resources, and effectively solving patients' health problems. The mastery of hypertension-related knowledge regarding hypertensive patients served by family doctors improved significantly; this can help patients master scientific and reasonable self-management methods, enhance self-care awareness, and implement behavior changes.

## 5. Conclusion

Diabetes and hypertension are the most common diseases and often coexist. Currently, hypertension is the most widespread chronic disease in China. In summary, the team's three-dimensional management under the medical community model significantly improves the ability of grassroot general practitioners to diagnose and treat hypertension and diabetes and better control diabetes and hypertension levels in patients.

Based on basic research concerning the standardized management intervention model for grassroot communities, this study provides innovation in exploring the three-dimensional management of teams within the grassroot medical community model. With the medical community model, community hospitals are closely and seamlessly connected to chronic diseases' three-dimensional management. The chronic disease management team trains the doctors in charge of the grassroot community about hypertension and diabetes, improves their diagnosis and treatment abilities, and effectively enhances the detection and treatment rates of hypertension and diabetes, thereby reducing the incidence of mortality through cardiovascular diseases. This model makes it more conducive to strengthen patients' education, including drug and nondrug treatment, emotional management, better management of blood pressure and blood glucose, and forming a good and healthy lifestyle, in order to improve patients' quality of life and provide an experimental basis to effectively control chronic diseases at the grassroot level. However, long-term follow-up observations are still lacking and need to be further explored in future studies.

## Figures and Tables

**Table 1:** Comparison of the basic situation of general practitioners in the study group and the control group.

Normal information	Research group (*n* = 59)	Control group (*n* = 59)	t/*χ*^2^	*p*
Age (years)	36.8 ± 7.2	37.4 ± 7.8	−0.434	0.665
Sex (%)				
Male	33 (55.93)	38 (64.41)	0.884	0.347
Female	26 (44.07)	21 (35.59)		
Job title (%)			1.221	0.229
Primary	33 (55.93)	27 (45.76)		
Intermediate	26 (44.07)	32 (54.24)		
Education (%)			2.365	0.307
College	17 (28.81)	10 (16.95)		
Undergraduate	38 (64.41)	44 (74.58)		
Postgraduate	4 (6.78)	5 (8.47)		

**Table 2:** Comparison of diabetes diagnosis and treatment ability before and after training.

Project	Research group (*n* = 59)	Control group (*n* = 59)	*χ* ^2^	*p*
Diagnosis of type 2 diabetes (%)				
Before training	36 (61.02)	39 (66.1)	0.329	0.566
After training	57 (96.61)	46 (77.97)	9.241	0.002
Impaired glucose tolerance (%)				
Before training	40 (67.8)	43 (72.88)	0.366	0.545
After training	55 (93.22)	50 (84.75)	2.161	0.142
Impaired fasting blood sugar (%)				
Before training	27 (45.76)	32 (54.24)	0.847	0.357
After training	57 (96.61)	46 (77.97)	9.241	0.002
HbA1c purpose (%)				
Before training	34 (57.63)	40 (67.8)	1.305	0.253
After training	58 (98.31)	50 (84.75)	6.993	0.008
Dyslipidemia characteristics (%)				
Before training	24 (40.68)	28 (47.46)	0.550	0.458
After training	49 (83.05)	40 (67.8)	3.703	0.054
Blood sugar control goals (%)				
Before training	25 (42.37)	30 (50.85)	0.851	0.356
After training	57 (96.61)	49 (83.05)	5.937	0.015
Drugs of choice for obese patients (%)				
Before training	26 (44.07)	32 (54.24)	1.221	0.269
After training	55 (93.22)	47 (79.66)	4.627	0.031
The drug of choice for nonobese patients (%)				
Before training	40 (67.8)	35 (59.32)	0.915	0.339
After training	56 (94.92)	50 (84.75)	3.340	0.068

**Table 3:** Comparison of the ability to diagnose and treat hypertension before and after training.

Project	Research group (*n* = 60)	Control group (*n* = 60)	*χ* ^2^	*p*
Blood pressure level classification (%)				
Before training	36 (61.02)	40 (67.8)	0.591	0.442
After training	58 (98.31)	50 (84.75)	6.993	0.008
Risk stratification (%)				
Before training	18 (30.51)	23 (38.98)	0.934	0.334
After training	48 (81.36)	40 (67.8)	2.861	0.091
Antihypertensive treatment strategies (%)				
Before training	26 (44.07)	21 (35.59)	0.884	0.347
After training	50 (84.75)	40 (67.8)	4.683	0.03
Reasonable diet (%)				
Before training	39 (66.1)	35 (59.32)	0.58	0.446
After training	55 (93.22)	50 (84.75)	2.161	0.142
Weight control (%)				
Before training	41 (69.49)	36 (61.02)	0.934	0.334
After training	56 (94.92)	50 (84.75)	3.34	0.068
Physical exercise (%)				
Before training	32 (54.24)	36 (61.02)	0.555	0.456
After training	57 (96.61)	52 (88.14)	3.007	0.083
Quit smoking (%)				
Before training	29 (49.15)	33 (55.93)	0.544	0.461
After training	51 (86.44)	47 (79.66)	0.963	0.326
Balance mind (%)				
Before training	22 (37.29)	18 (30.51)	0.605	0.437
After training	53 (89.83)	43 (72.88)	5.587	0.018
Cautionary use of diuretics (%)				
Before training	22 (37.29)	26 (44.07)	0.562	0.453
After training	48 (81.36)	40 (67.8)	2.861	0.091
Caution/prohibition of *ß* blockers (%)				
Before training	26 (44.07)	23 (38.98)	0.314	0.575
After training	50 (84.75)	42 (71.19)	3.157	0.076
ACEI drug prohibition certificate (%)				
Before training	22 (37.29)	27 (45.76)	0.873	0.35
After training	52 (88.14)	45 (76.27)	2.978	0.084
Caution/prohibition of compound preparation (%)				
Before training	17 (28.81)	23 (38.98)	1.362	0.243
After training	50 (84.75)	40 (67.8)	4.683	0.040

**Table 4:** Comparison of baseline data of patients in the study group and the control group with general practitioner intervention.

Normal information	Research group (*n* = 200)	Control group (*n* = 200)	t/*χ*^2^	*p*
Age (years)	70.5 ± 6.7	69.4 ± 6.7	1.642	0.101
BMI (kg/m^2^)	24.8 ± 1.9	24.5 ± 2.3	1.422	0.156
Course of disease (years)	7.2 ± 2.2	7.0 ± 2.0	0.951	0.342
Sex (%)			0.493	0.483
Male	111 (55.5)	104 (52.00)		
Female	89 (44.5)	96 (48.00)		
Disease (%)			0.812	0.368
Hypertension	100 (50.00)	109 (54.5)		
Diabetes	100 (50.00)	91 (45.5)		
Smoking (%)			0.433	0.511
Yes	56 (28.00)	62 (31.00)		
No	144 (72.00)	138 (69.00)		
Drinking (%)			0.552	0.468
Yes	70 (35.00)	63 (31.5)		
No	130 (65.00)	137 (68.5)		
Hyperlipidemia (%)			0.57	0.458
Yes	59 (29.5)	66 (33.00)		
No	141 (70.5)	134 (67.00)		
Coronary heart disease (%)			1.567	0.211
Yes	26 (13.00)	32 (16.00)		
No	174 (87.00)	168 (84.00)		

**Table 5:** Blood pressure control status of study group and control group.

Group	*n*	SBP (mmHg)		DBP (mmHg)	
		Before intervention	After intervention	Before intervention	Afterintervention
Research group	100	157.2 ± 8.6	128.0 ± 7.0	98.4 ± 6.6	76.1 ± 5.8
Control group	109	155.5 ± 8.1	131.4 ± 6.7	97.0 ± 7.0	77.6 ± 6.3
*t*		1.472	-3.587	1.484	−1.786
*p*		0.143	0.000	0.139	0.076

**Table 6:** The blood sugar control status of the study group and the control group$\left(\bar{x}\pm s\right)$.

Group	*n*	FPG (mmol/L)		2hPG (mmol/L)		HbA1c (%)	
		Before intervention	After intervention	Before intervention	After intervention	Before intervention	After intervention
Research group	100	8.84 ± 0.95	6.32 ± 0.55	12.78 ± 1.33	8.17 ± 1.05	8.86 ± 0.95	6.81 ± 0.68
Control group	91	8.70 ± 0.90	6.47 ± 0.67	12.51 ± 1.20	8.50 ± 1.23	8.64 ± 0.89	7.25 ± 0.74
*t*		1.043	-1.697	1.468	-1.999	1.647	-4.282
*p*		0.298	0.091	0.144	0.047	0.101	0.000

**Table 7:** Comparison of compliance between the study group and the control group [n(%)]..

Group	*n*	Complete compliance	General	Poor compliance
Research group	200	134 (67.00)	54 (27.00)	12 (6.00)
Control group	200	105 (52.50)	71 (35.50)	24 (12.00)
*Z*		−3.107		
*p*		0.002		

## Data Availability

The simulation experiment data used to support the findings of this study are available from the corresponding author upon request.
